# Empirical Analysis of Financial Depth and Width Based on Convolutional Neural Network

**DOI:** 10.1155/2021/8650059

**Published:** 2021-12-02

**Authors:** Mengqi Ye, Lijun Zhang

**Affiliations:** ^1^Zhejiang Agricultural Business College, Shaoxing, Zhejiang 312000, China; ^2^School of Management, Hebei Geo University, Shijiazhuang, Hebei 050031, China

## Abstract

There are great differences in financial and economic development in different regions. In different time series and different regions, the effects of financial depth and width on economic development are also different. This paper selects neural network to establish the economic benefit model of financial depth and breadth, which can deeply explore the relationship between financial data and economic data. In order to determine the optimal convolutional neural network parameters, the optimal convolutional neural network parameters are determined through comparative simulation analysis. The convolutional neural network model based on the optimal parameters is applied to the empirical analysis of the effect of financial and economic development in *X* region. In order to obtain the optimal convolutional neural network parameters, different convolution layers, convolution core size, and convolution core number are compared and simulated. The convolutional neural network model with optimal parameters is used to simulate the financial and economic data of *X* region. The simulation results show that the density of financial personnel has a certain impact on economic development, so it is necessary to improve the comprehensive quality of financial personnel and promote regional economic development. Therefore, this paper seeks an effective method to study the effect of financial breadth and depth on economic development which can provide a feasible idea for the in-depth research method of financial and economic development.

## 1. Introduction

In the development of China's market economy, people have conducted continuous and in-depth research on the relationship between financial development and economic growth [1]. However, in the existing studies, there are often different conclusions about the relationship between the two [2]. According to the relevant literature research, we can see that (1) in different stages of economic development, there will be considerable differences in the financial structure of nonpass regions. (2) Financial development is a complex concept with many connotations, and there will be great differences in the selection of measurement indicators [3]. (3) Everyone is trying to find an optimal matching; it is difficult to achieve this goal [4]. Chen et al. analyzed taking the financial depth scale and relevant financial indicators as independent variables. Therefore, it is suggested to increase the financial scale of banking industry and government intervention [5]. Feng et al. proposed the relationship between the financial system and financial development. Financial integration is regarded as a key indicator to adapt to the relevance of different market segments and realize the complementary relationship in finance [6].

Acedański et al. found that financial development has a significant impact on economic growth by studying the financial development in 1996. It can also stimulate economic growth through technological innovation [7]. Khan et al. discussed the influence of national culture dimension on financial development [8]. Chen et al. discussed the impact of capital flows on the financial development of some African countries from 1999 to 2014 and examined the relationship between two different forms of capital flows and economic development. Without considering financial development and human capital measures, FDI will have inhibitory effect on financial development and human capital [9]. Nasir et al. used fixed effect and generalized method of moments to conduct a study on regional effect and Asian economy. The results show that market-oriented development has a significant positive impact on the development of regional finance [10]. In the study of financial and economic development, Nasir et al. also introduced carbon emission indicators. Based on the data of 36 years from 1980 to 2016, they discussed that the long-term and short-term impact of a country trade openness and financial development on the national economy is negative and nonmaterial [11]. In the existing empirical analysis, it is difficult to draw a general conclusion on the interaction between financial development and economic growth, especially on the influencing factors of economic development in the transitional countries. Niranjan et al. studied the economies during the transition period, analyzed the relationship between financial development and economic growth, and analyzed the economic data of Southeast European countries by using the frequency Granger causality test method [12]. The analysis is conducive to sorting out the relevant factors with positive significance for economic development, so as to provide decision support for the country to put forward corresponding strategies, which is of great significance for the development of national economy [13].

The main method used in this research is the improved convolutional neural network technology to realize the deep mining and prediction analysis of financial data [13]. In the field of deep learning, convolutional neural network has achieved great success in image, video, and speech recognition and other fields. Convolutional neural network can be divided into one-dimensional, two-dimensional, and three-dimensional convolutional neural network according to its network structure, which can recognize medical image and video data [14]. Convolutional neural network has a very good performance in various industries, because of its excellent performance; it has a very good application effect in image classification and counting. Suma et al. designed a new automatic financial recognition method using deep convolutional neural network, which can achieve high-performance financial image classification [15]. Todd used convolutional neural network to recognize posture changes and combined with local binary pattern recognition to realize face image recognition [16]. In biomedical engineering applications, Todd et al. proposed the method of using convolutional neural network to accurately detect QOS wave group. CNN method can extract ECG morphological features of different granularity, so as to realize a simple and practical ECG signal prediction processing technology. In practical application, this method can achieve 99.77% sensitivity and accuracy [16].

As the innovation and development of the financial field, the market environment plays a very important role in green finance. Williams et al. proposed a deep learning model based on convolutional neural network to build a green intelligent financial system, which realized the cleaning of financial data and the extraction of data structure. The concurrent model has good system robustness [17]. This research will build an index system covering the width and depth of finance to ensure the scientificity and integrity of the evaluation index system. Secondly, by using the method of empirical analysis, we can understand their growth effects and grasp the overall trend of economic growth and financial growth. The connotation of the relevant index data can be deeply mined, which can provide countermeasures and suggestions for economic development based on the characteristics of financial development in different regions.

In order to find an effective method to study the impact of financial breadth and depth on economic development, it can provide a feasible idea for the in-depth research method of financial and economic development. This paper creatively selects neural network to establish the economic benefit model of financial depth and breadth, which can deeply explore the relationship between financial data and economic data. In order to determine the optimal convolutional neural network parameters, the optimal convolutional neural network parameters are determined through comparative simulation analysis. The convolutional neural network model based on the optimal parameters is applied to the empirical analysis of the effect of financial and economic development in *X* region. In order to obtain the optimal convolutional neural network parameters, different convolution layers, convolution kernel size, and convolution kernel number are compared and simulated. The convolutional neural network model based on the optimal parameters is applied to the empirical analysis of the effect of financial and economic development in *X* region. Through simulation analysis, financial breadth index (insurance density, financial institution density, and financial personnel density) and financial depth index (insurance depth, monetization degree, and securitization degree) and economic benefit index are analyzed.

This paper is divided into five parts. The first part expounds the research background. There are great differences in financial and economic development in different regions. In different time series and different regions, the impact of financial depth and width on economic development is also different. The second part describes the optimization and improvement of BP neural network and convolutional neural network. The third part analyzes the economic growth effect of financial depth and width based on convolutional neural network. The fourth part studies the impact of financial depth and width on economic growth and constructs an economic benefit model based on convolutional neural network. Finally, the results are analyzed and the effects of different convolution parameters on the prediction difference are summarized.

## 2. Artificial Neural Network

Artificial neural network is an algorithm model that simulates the propagation mechanism of biological neural system. It can use a large number of simulated neurons to realize the propagation of information and deeply explore the internal complex relationship between data. In the artificial neural network, the most basic information transmission unit is called neuron. The neuron uses the activation function to map a large number of neural network inputs and amplifies or suppresses them to achieve the set output goal. A typical artificial neuron is shown in Figure 1.

Let the input of the *n*th neuron be *x*_*n*_, the output neuron be *y*, the connection weight of the input value be *w*_*n*_, and the threshold be *θ*,

(1) $$\begin{array}{c} y=f\left(\sum_{j=1}^{n}w_{j}x_{j}-\theta \right). \end{array}$$

There are five common types of activation functions, which are step function, linear function, saturated linear function, S-type function, and Gaussian function.

If only a single neuron is applied, it can only solve some simple problems. For complex tasks, it must be based on a complex neural network composed of a single neuron. They can be divided into interconnected network structure and hierarchical network structure.

The topological structure of hierarchical neural network is shown in Figure 2. Different structures are connected by multiple neurons to form a complete artificial neural network. All the results are output through the output layer network. The internal processing part of neural network is hidden layer, through which neural network can realize deep learning and data feature extraction.

The difference between interconnected neural network and hierarchical neural network is that it can take the output of lower neurons as the input data of upper neurons. The most common interconnected neural networks are Hopfield network and Boltzmann machine network (Figure 3).

## 3. BP Neural Network

BP neural network is a kind of multilayer neural network that adjusts each layer based on the connection weight, so as to form the BP network structure diagram. Let the input vector be *X*, the output vector be *Y*, the target output vector be *d*=(*d*_1_, *d*_2_,…,*d*_*l*_)^*T*^, the output vector of the output layer be *O*=(*o*_1_, *o*_2_,…,*o*_*l*_)^*T*^, the connection weight matrix of the input layer and the hidden layer be *V*=(*V*_1_, *V*_2_,…, *V*_*m*_), and the link weight of the *j*^th^ neuron be *V*_*j*_. In BP neural network, the activation function is expressed as

(2) $$\begin{array}{c} O_{k}=f\left(u_{k}\right),\;k=1,2,\ldots ,l. \end{array}$$

The input layer of BP neural network is as follows:

(3) $$\begin{array}{c} \Delta v_{ij}=\eta .\delta_{j}^{y}.x_{i}=\eta .\left(\sum_{k=1}^{l}\delta_{k}^{o}.w_{jk}\right).y_{j}.\left(1-y_{j}\right).x_{i}. \end{array}$$

The activation function of the hidden layer is expressed as

(4) $$\begin{array}{c} u_{j}=\sum_{i=0}^{n}v_{ij}\cdot x_{i},\;j=1,2,\ldots ,m. \end{array}$$

Here, we select sigmoid function, which is continuously differentiable,

(5) $$\begin{array}{c} f\left(x\right)=\frac{1}{1+e^{-x}}, \end{array}$$

corresponding to

(6) $$\begin{array}{c} f\left(x\right)=f\left(x\right)\left[1-f\left(x\right)\right]. \end{array}$$

The output error can be defined as

(7) $$\begin{array}{c} E=\frac{1}{2}{\left(d-O\right)}^{2}=\frac{1}{2}\sum_{k=1}^{l}{\left(d_{k}-O_{k}\right)}^{2}. \end{array}$$

Substituting equation (7) into the output layer, we can get the following results:

(8) $$\begin{array}{c} E=\frac{1}{2}{\sum_{k=1}^{l}\left[d_{k}-f\left(\sum_{j=0}^{m}w_{jk}.y_{j}\right)\right]}^{2}. \end{array}$$

By expanding it to the hidden layer, we can get the following results:

(9) $$\begin{array}{c} E=\frac{1}{2}{\sum_{k=1}^{l}\left\{d_{k}-f\left[\sum_{j=0}^{m}w_{jk}.f\left(\sum_{l=0}^{n}v_{ij}.x\right)\right]\right\}}^{2}. \end{array}$$

In order to reduce the error value,

(10) $$\begin{array}{c} \Delta w_{jk}=-\eta .\frac{\partial E}{\partial w_{jk}},\;j=0,1,2,\ldots ,m,\;k=1,2,\ldots ,l. \end{array}$$

(11) $$\begin{array}{c} \Delta w_{jk}=-\eta .\frac{\partial E}{\partial w_{ij}},\;i=0,1,2,\ldots ,n,\;j=1,2,\ldots ,m. \end{array}$$

In equations (10) and (11), “−” denotes gradient descent. *η* is a constant in the range of (0, 1), which represents the learning rate.

By adjusting the connection weights of equations (10) and (11),

(12) $$\begin{array}{c} \delta_{k}^{o}=\frac{\partial E}{\partial u_{k}}=-\frac{\partial E}{\partial o_{k}}.\frac{\partial o_{k}}{\partial u_{k}}=-\frac{\partial E}{\partial o_{k}}.f\prime \left(u_{k}\right),\\ \delta_{j}^{y}=\frac{\partial E}{\partial u_{j}}=-\frac{\partial E}{\partial o_{j}}.\frac{\partial o_{j}}{\partial u_{j}}=-\frac{\partial E}{\partial o_{j}}.f\prime \left(u_{j}\right). \end{array}$$

From equation (7), it can be obtained that

(13) $$\begin{array}{c} \frac{\partial E}{\partial O_{k}}=-\left(d_{k}-O_{k}\right),\\ \frac{\partial E}{\partial y_{j}}=-\sum_{k=1}^{l}\left(d_{k}-O_{k}\right)\cdot f^{\prime }\left(u_{k}\right)\cdot w_{jk}. \end{array}$$

Furthermore, we can get the following results:

(14) $$\begin{array}{c} \delta_{k}^{o}=\left(d_{k}-O_{k}\right).O_{k}.\left(1-O_{k}\right),\\ \delta_{j}^{y}=\left[\sum_{k=1}^{l}\left(d_{k}-O_{k}\right).f^{\prime }\left(u_{k}\right).w_{jk}\right].f^{\prime }\left(u_{j}\right). \end{array}$$

Namely,

(15) $$\begin{array}{c} \delta_{j}^{y}=\left(\sum_{k=1}^{l}\delta_{k}^{o}.w_{jk}\right).y_{j}.\left(1-y_{j}\right). \end{array}$$

In this way, the error calculation formula of output layer and hidden layer can be deduced:

(16) $$\begin{array}{c} \Delta w_{jk}=\eta .\delta_{k}^{o}.y_{j}=\eta .\left(d_{k}-O_{k}\right).O_{k}.\left(1-O_{k}\right).y_{j},\\ \Delta v_{ij}=\eta .\delta_{j}^{y}.x_{i}=\eta .\left(\sum_{k=1}^{l}\delta_{k}^{o}.w_{jk}\right).y_{j}.\left(1-y_{j}\right).x_{i}. \end{array}$$

## 4. Optimization and Improvement of Convolutional Neural Network

Convolutional neural network was first proposed by Hubel and another biologist in 1962. Then, it was introduced into neural network by Fukushima to form neural perceptron. Finally, BP algorithm was used to train convolutional neural network. Convolutional neural network was originally used in handwritten character recognition. Local feature extraction and transformation can be carried out among the neurons, and the neurons with the same connection weight can be connected with the upper layer neural network region to form a parallel neural network structure with invariable properties.

The typical calculation process of convolutional neural network is shown in Figure 4. A convolution layer often contains multiple feature mapping surfaces and the neurons in the feature mapping surface. The neurons in each feature mapping surface only receive the propagation information of the receiving domain. The next layer of convolution layer is downsampling layer. Convolution layer and downsampling layer appear almost at the same time. The downsampling layer can reduce the number of free parameters, reduce the output deformation sensitivity, and then reduce the computational complexity of neural network [18].

Before the network training, the connection weights are set to different random numbers, and then the forward and backward propagation network training is carried out. In the network training of forward propagation, let the input of the network be *X*. The output formula of the output layer is as follows after the input information is calculated layer by layer:

(17) $$\begin{array}{c} O_{p}=F_{n}\left(\cdots \left(F_{2}\left(F_{1}\left(XW_{1}\right)W_{2}\right)\cdots \right)W_{n}\right). \end{array}$$

Let the error of network training result be *E*_*p*_, i.e., the difference between *O*_*p*_ and *Y*_*p*_; the equation is

(18) $$\begin{array}{c} Ep=\frac{1}{2}{\left(y_{pj}-o_{pj}\right)}^{2}. \end{array}$$

Convolution in convolutional neural network includes effective convolution and invalid convolution. Let the two lengths be *L*_1_, *L*_2_, respectively. In the process of information propagation, convolution kernel uses effective convolution to realize forward propagation. Let the degree of downsampling be *s* that the downsampling layer will copy a total of *s*^2^ errors and then sigmoid the errors. The reverse propagation process of convolution is to rotate the convolution kernel 180° to convolute the convolution kernel and the error completely. Calculate the connection relationship between the upper feature mapping layer and the current feature mapping layer and update the connection weight by convolution.

In convolutional neural network, each network parameter is trained and learned by samples first, and useful features can be obtained from training samples after training. The sharing of connection weight improves the network efficiency. In convolutional neural network, the input of delayed neurons is less, which makes the number of layers of propagation gradient network increase. The prior structure between the two layers is also very suitable for pattern recognition. As long as we can select an appropriate value range before network training, we can ensure that the network can get a good training effect.

## 5. Analysis of Economic Growth Effect of Financial Depth and Width Based on Convolutional Neural Network

### 5.1. Economic Growth Effect of Financial Depth and Width

The impact of financial development on the economy can be analyzed from the two dimensions of financial width and depth. Financial development has an impact on the economy based on these two dimensions, and economic growth will have an impact on financial development. This relationship is shown in Figure 5.

From the perspective of capital supply and demand, in the demand-oriented market, the development of the product market will continue to promote the expansion of the market. In this process, the risk can be effectively dispersed, so as to achieve the control of transaction costs. In the process of market expansion, the demand for capital is also increasing [19]. The improvement of TFP is the result of the development of economic sectors, which can show the role of financial system in promoting economic growth, which is a passive role. In the supply-oriented market, the financial deepening in financial development has become an independent variable, and the resources in the financial system will be transferred to some financial deepening departments, so as to promote the growth of resources by providing more resources for those more dynamic projects. Generally speaking, the process of financial development is from supply-oriented to demand-oriented financial system and gradually tends to be mature [20].

From the perspective of credit, financial institutions will maintain a more cautious attitude when providing loans to nonstate-owned enterprises. From the perspective of actual production and case analysis, the marginal productivity of credit capital of nonstate-owned enterprises is more than that of state-owned enterprises, and there will be a significant resource tilt in the allocation of financial resources of state-owned enterprises; state-owned enterprises can increase output and produce economic benefits while enjoying more resources. From the perspective of monetization, when the government implements a more relaxed and active monetary policy, the domestic credit business will have a positive effect on the economic contribution. When the government implements a tighter monetary policy, its contribution to economic development will decline. This is because the mode of economic growth is an extension expansion.

From the perspective of spatial distribution, financial development is a kind of regional and organizational agglomeration. The development of financial sector is inseparable from the distribution of social resources. Modern financial development has long been free from the labor-intensive characteristics and has become a highly technology intensive economic activity. The maturity of any financial system requires highly skilled talents. When the opportunity cost of human capital exceeds the cost of financial activities, it will hinder the long-term economic growth. From the perspective of insurance market, the insurance industry can play a positive role in supporting the stable development of social economy, expanding investment and stimulating consumption and playing a positive role in people's life and economic trade.

Three indicators of financial depth are determined, namely, insurance depth, monetization degree, and securitization degree, and three indicators of financial width are determined, namely, insurance density, financial institution density, and financial personnel density.

### 5.2. Economic Benefit Model Construction Based on Convolutional Neural Network Financial Depth and Width

The subject matter covered by in-depth research is limited and the tracking time is long, which is more suitable for the long-term odds first trading system. Breadth research covers many subjects, so it is necessary to judge the winning rate of investment subjects first. Therefore, there are many financial depth and breadth indicators. In order to be applied to convolutional neural network, we set up comprehensive indicators of financial depth and breadth and comprehensive indicators of economic benefits for analysis. The time series of finance makes the value of financial development change all the time. By analyzing the historical value of financial development in a certain period, we can predict and analyze its impact on economic development benefits. Select sliding window technology to extract data units from historical data.

Let the sample length of convolutional neural network model be *l* and the downsampling amplitude be *s*.

(19) $$\begin{array}{c} \frac{\left[\left(l-c+1\right)/s-c+1\right]}{s}=N. \end{array}$$

For single-layer convolution and downsampling, equation (20) is satisfied as follows:

(20) $$\begin{array}{c} \frac{\left(l-c+1\right)}{s}=N. \end{array}$$

In equation (20), for financial data, due to the impact of time series, the impact on financial time series data at a certain time will directly affect the length of the sample. For different sample lengths, the range of convolution kernel size is shown in Table 1.

In order to realize the analysis and research of neural network in financial and economic benefits, data preprocessing, parameter initialization, model training, and data output are needed. In order to train and test different financial time series data, it is necessary to initialize the data.

For a large number of financial data, there may be abnormal or missing data. Therefore, preprocessing is needed before data processing, including data cleaning and transformation. The noise, abnormal value, and missing value in the original data are removed. Data transformation adopts normalization, dimension reduction, and other measures. The abnormal data value is mainly for the data less than 0. The most typical one is kernel smoothing method. At present, it is widely used in the analysis and prediction of financial time series and can have good denoising effect.

Let the kernel function be *K*_*h*_(*x*), the time series of financial data be {*Y*_*t*_}, the coordinates of the sample center point *Y*_*t*_ be *X*_*t*_, and the processed sequence value of {*Y*_*t*_} be *m*_*h*_(*x*). The kernel function is used to distribute the weight of observation data points.

(21) $$\begin{array}{c} m_{h}\left(x\right)\frac{\sum_{t=1}^{T}K_{h}\left(x-X_{1}\right)Y_{t}}{\sum_{t=1}^{T}K_{h}\left(x-X_{t}\right)},\\ K_{h}\left(x\right)=\frac{1}{h\sqrt{2\pi }}e^{-x^{2}/2h^{2}}. \end{array}$$

The larger the data of financial time series is, the less conducive it is to the calculation of the model, so we need to use the normalization method to unify the data in a range. The selected text data is placed in [0, 1]. Suppose that the time series of financial data is {*Y*_*t*_}, the time series value of time *t* is *y*_*t*_, and the maximum and minimum values of the time series are max{*Y*_*t*_}, min{*Y*_*t*_}, respectively.

(22) $$\begin{array}{c} y_{t}^{\prime }=\frac{y_{t}-\min\left\{Y_{t}\right\}}{\max\left\{Y_{t}\right\}-\min\left\{Y_{t}\right\}}. \end{array}$$

## 6. Results Analysis

### 6.1. Influence of Different Convolution Parameters on Prediction Difference

In order to determine the best number of convolution layers. The simulation test results are shown in Figures 6 and 7, respectively.

It can be seen calculated are better than those calculated when the convolution level is 1, but the difference is small. In the empirical analysis, it is more reasonable to set the convolution level as 2.

Through the analysis of Figures 8 and 9, it is determined that the convolution kernel size is set to 3.

The influence of different convolution kernel numbers on the prediction results is shown in Table 2.

It can be seen from Table 2 that with the increase of the number of convolution kernels, the prediction results show a most reasonable and effective simulation results.

### 6.2. Empirical Analysis

Financial analysis is to analyze the financial benefits and costs of the project from the perspective of the interests of enterprises or investors. Economic analysis is to analyze the benefits and costs of the project to the whole national economy and even the whole society from the perspective of a country or region. This paper selects the financial data and economic-related data of area *X* for simulation analysis. According to the simulation analysis of financial width index (insurance density, financial institution density, and financial personnel density), financial depth index (insurance depth, monetization degree, and securitization degree), and economic benefit index, it judges the influence of each index on economic benefit. The details are shown in Figure 10.

In Figure 10, in the economic development of area *X*, financial breadth and financial depth show a consistent development trend. The density of financial personnel shows a regression effect to some extent, while the density of financial institutions shows a positive effect. From a comprehensive analysis, in order to achieve better economic growth benefits in *X* region, it is necessary to improve the quality of financial industry practitioners, rather than simply increasing the number of personnel, to ensure the quality of regional teaching and cultivate more high-quality financial personnel.

## 7. Conclusion

This paper selects neural network to build the economic benefit model of financial depth and width, which can deeply mine the relationship between financial data and economic data. In order to determine the best convolutional neural network parameters, through comparative simulation analysis, the best convolutional neural network parameters are determined: convolution layer number is 2, convolution core size is 19, and convolution core numbers are 5 and 10. The convolutional neural network model based on the best parameters is applied to the empirical analysis of the effect of financial and economic development in *X* region. Through simulation, this paper analyzes the financial width index (insurance density, financial institution density, and financial personnel density), financial depth index (insurance depth, monetization degree, and securitization degree), and economic benefit index. The results show that, except for the density of financial personnel, the other indicators have played a positive role in the economic benefit growth of *X* region. In order to improve the economic growth efficiency of *X* region, we should improve the average quality of financial personnel and give full play to human resources. Compared with the traditional research methods, the algorithm proposed in this paper can deeply mine the relationship between financial data and economic data. In order to determine the optimal convolutional neural network parameters, the convolutional neural network model with the optimal parameters can provide more stable economic benefits in empirical analysis. In this study, only six typical indicators are selected to represent the width and depth of finance, but the financial indicators are complex, and more comprehensive indicators can be selected for more in-depth analysis in future research.

## Figures and Tables

**Figure 1:** Typical structure of artificial neuron.

**Figure 2:** The topological structure of hierarchical neural network.

**Figure 3:** The topological structure of interconnected neural network.

**Figure 4:** Calculation process of typical convolutional neural network.

**Figure 5:** The effect of different financial development dimensions on economic growth.

**Figure 6:** Simulation results with 1 convolution layer.

**Figure 7:** Simulation results with 2 convolution layers.

**Figure 8:** Simulation results when convolution kernel size is 3.

**Figure 9:** Simulation results when convolution kernel size is 19.

**Figure 10:** Empirical simulation analysis.

**Table 1:** Relationship between sample length and convolution kernel size.

Input sample length	30	40	50	60
Convolution kernel size range	7	13	15	17
	3	9	11	13
	-	5	7	9
	-	-	3	5

**Table 2:** Analysis of the influence of different convolution kernel numbers on prediction results.

Number of convolution kernels	(3, 6)	(4, 8)	(5, 10)	(6, 12)
Root mean square error	6.8947	6.8532	6.1146	6.5236
Correlation coefficient	0.8992	0.8975	0.8883	0.8841
Coefficient of certainty	1.0314	1.0526	1.0018	0.9659

## Data Availability

The data used to support the findings of this study are available from the corresponding author upon request.
